# Clinical Image Feature Analysis and Diagnostic Efficacy Evaluation of Pulmonary Ultrasound in the Diagnosis of Congenital Pulmonary Airway Malformations in Children: Based on a Single Center, Retrospective Cohort Study

**DOI:** 10.1155/2022/7490207

**Published:** 2022-08-18

**Authors:** Dandan Liu, Gang Zhang, Jianyi Liao, Lan Jiang, Chun Cai, Xiao Li, Lei Lou, Bin Zhou, Huiyi Zeng, Xiangang Yan, Gang Yu

**Affiliations:** ^1^Department of Ultrasound Medicine, The Third Affiliated Hospital of Guangzhou Medical University, Guangzhou, China; ^2^Department of Pediatric Surgery, The Third Affiliated Hospital of Guangzhou Medical University, Guangzhou, China

## Abstract

**Objective:**

A single center, retrospective cohort study was conducted to analyze the clinical image features and diagnostic efficiency of pulmonary ultrasound in the diagnosis of congenital pulmonary airway malformations (CPAMs) in children.

**Methods:**

The starting and ending time of this study is from May 2019 to December 2021. This study included 200 children with CPAM diagnosed by prenatal ultrasound and postpartum CT imaging (aged from 1 hour to 3 years), including 103 males and 97 females. All of them were diagnosed by fetal ultrasound and were examined by chest X-ray (CXR), chest CT, and lung ultrasound (LUS). The clinical image characteristics and diagnostic efficiency of CXR, chest CT, and LUS in the diagnosis of CPAM in children were analyzed.

**Results:**

200 lesions were limited to single lung, and the most common were right lower lobe, right lower lobe in 80 cases (40.0%), left lower lobe in 60 cases (30.0%), right upper lobe in 30 cases (15.0%), left upper lobe in 20 cases (10.0%), and right middle lobe in 10 cases (5.0%). Among the 200 cases of preoperative CT examination, 196 cases (98.00%) showed lesions and confirmed diagnosis, and 4 cases were missed. Chest X-ray showed multiple focal circular low-density shadow in the right lung, and the heart shadow and mediastinum moved slightly to the left. CXR showed multiple cystic transparent shadows in the left lower lung and slightly to the right of the mediastinum and heart. CXR showed multiple balloon cavities of different sizes in the right lung field, and the mediastinum and heart shadow shifted to the left. The direct signs of LUS (including single or multiple cystic lesions) were not significantly different from those of CXR, but the indirect signs were significantly higher than those of CXR.

**Conclusion:**

The most common CT findings of CPAM in children are cystic lesions, especially polycystic lesions, while LUS images of CPAM in children are various. LUS is a noninvasive and nonradiological examination method, which is easy to operate and repeat. LUS can be used for preliminary qualitative screening of CPAM in children, and the diagnostic value of indirect signs of LUS is better than that of CXR.

## 1. Introduction

Congenital pulmonary airway malformation (CPAM) is a congenital pulmonary dysplasia of unknown etiology. The essence of this disease is large airway obstruction and pulmonary parenchyma dysplasia. This malformation often occurs in the early stage of lung embryonic development [1]. In 1977, Tian et al.[2] divided the disease into types I, II, and III according to the clinical and pathological features. In 2002, An et al. [3] changed the name of CCAM to CPAM and changed the original three-point method to a five-point method which was divided into 0–4 types according to the different parts of the airway where the malformations occurred. The latter two are widely used in clinic. CPAM is a hamartoma-like lesion characterized by a polycystic mass of lung tissue with abnormal bronchial proliferation. Its incidence is 10410 000, which is slightly higher in men, often involving part of the lung lobe or the whole lobe. 80% of the lesions are located in a single lobe, and about 1% of the lesions occur in the bilateral lobes [3]. The clinical manifestations of the CPAM are generally dyspnea, fever, cough, and other nonspecific symptoms; some cases may also be asymptomatic. It has been reported in previous literature that the disease can be secondary to malignant tumors such as adenocarcinoma and squamous cell carcinoma. In addition, some cases are pathologically difficult to distinguish from low-grade pleural pulmonary blastoma (PPB) [4], so lobectomy is recommended no matter whether it is symptomatic or not. Because the clinical manifestations and laboratory results of CPAM are not specific, its diagnosis mainly depends on imaging examination, so it is necessary to study the imaging manifestations of CPAM.

With the development of prenatal ultrasound imaging technology, most CPAM can be diagnosed in the fetal period. It is reported in the literature that most of the children with CPAM have a good prognosis, and about 5% of them have respiratory symptoms after birth, which need to be diagnosed as soon as possible and surgical intervention should be carried out in time. Children who are asymptomatic after birth but those whose chest lumps are revealed by ultrasound often face a series of postpartum chest X-rays. When their CXR test is negative, they may also need to undergo chest enhanced CT for imaging diagnosis [5]. In addition, for children with twins or multiple births with CPAM, twins or even multiple births may need to be diagnosed by CXR or even chest enhanced CT. Lung ultrasound (LUS), as an important examination and therapeutic effect monitoring method for the diagnosis of lung diseases, has been successfully used to diagnose a variety of neonatal lung diseases, such as respiratory distress syndrome, wet lung, pulmonary hemorrhage, pneumonia, atelectasis, meconium aspiration syndrome, and pneumothorax. At present, although there are many reports about prenatal ultrasound diagnosis of CPAM, there is less literature about the ultrasonographic features of neonatal CPAM [6]. In this study, the clinical data of 200 children with CPAM were retrospectively analyzed, the ultrasonographic features of CPAM in neonatal period were summarized, the accuracy of CXR and LUS in the diagnosis of congenital pulmonary airway malformation was compared, and the clinical diagnostic value of neonatal LUS in CPAM was discussed. In this paper, the clinical image characteristics and diagnostic efficiency of LUS in the diagnosis of CPAM in children were analyzed retrospectively, in order to improve the understanding and diagnostic accuracy of the disease.

## 2. Patients and Methods

### 2.1. Patients Information

The starting and ending time of this study is from May 2019 to December 2021. This study included 200 children with CPAM diagnosed by prenatal ultrasound and postpartum CT imaging (aged from 1 hour to 3 years), including 103 males and 97 females. All the children were diagnosed by fetal ultrasound and were examined by CXR, chest CT, and LUS. This study was approved by the Medical Ethics Association of our hospital, and all patients signed informed consent.

### 2.2. Investigation Methods

Chest CT examination: Siemens FROCE dual-source 194 layer ct, scanning range from the top of the chest entrance to the bottom of the lung, scanning parameters: plain scan tube voltage 120 kV, tube current 27 mAs. Dual-source scanning was used, including A ball tube voltage 70 kV, tube current 30–35 mAs tube voltage 150 kV, tube current 11–15 mAs, matrix 25 cm tube 25 cm, conventional slice thickness 3 mm and 0.6 mm thick lung window image, nonionic iodine contrast medium enhanced examination, nurse hand injection, and dose of 1.5 ml/kg.

LUS examination: using HITACHI ALOKA and PHILIPS ultrasonic diagnostic instrument, high frequency linear array probe, frequency 8–12 MHz. The LUS examination of the children was performed by two attending physicians who had received special lung ultrasound training. In the quiet state, the supine position, lateral position, and prone position were taken, and each lung was divided into three regions: anterior, lateral, and posterior regions, that is, 6 regions on both sides of the chest, which were bounded by the parasternal line, anterior axillary line, posterior axillary line, and spinal line on both sides of the chest, and each side of the lung was divided into three regions: the anterior area, the lateral area, and the posterior area, that is, six regions on both sides of the lungs. Each region of the lung needs to be scanned longitudinally (the probe is perpendicular to the ribs) and transversely (the probe walks along the intercostal space), and each region is scanned one by one from top to bottom, the order of which is, first, check the anterior area of the chest, the range between the parasternal line and the anterior axillary line; then check the lateral area of the chest, the range between the anterior axillary line and the posterior axillary line; finally, check the posterior area of the chest, the range between the posterior axillary line and the spinal line [7]. LUS observation index: direct signs included anechoic cystic lesions, high echo area, and low echo area, indirect signs included abnormal pleural line, A-line, B-line, pulmonary consolidation with bronchial inflation sign, pleural effusion, and mediastinal displacement.

CXR inspection: use GE1 instead of DR camera to shoot, and upload to Tianjian PACS system to read the film. The direct signs of X-ray findings included liquid cysts, gas-liquid cysts, air cysts, and multiple pulmonary cysts, while the indirect signs included emphysema, pulmonary consolidation, exudative lesions, and mediastinal displacement.

### 2.3. Image Analysis

The preoperative imaging data of all cases were collected retrospectively, including chest CT imaging diagnosis and images, CXR, and LUS imaging diagnosis and images. The imaging diagnosis was completed by two imaging doctors, one of whom had more than 10 years of work experience. The imaging data included the location of the lesion, the extent of involvement, the shape of the lesion and its surrounding manifestations, and whether there was systemic blood supply.

### 2.4. Statistical Analysis

SPSS 19.0 software was used for statistical analysis, the measurement data were expressed as $\bar{x}\pm s$, the counting data were expressed as constituent ratio (%), and the Fisher exact probability method was used for comparison between groups. *T*-test and *χ*^2^ test were used to compare the two groups, and *P* < 0.05 indicates that there is significant difference between the two groups.

## 3. Results

### 3.1. Diagnosis Result

All the 200 lesions were confined to the single lung lobe, most commonly in the lower lobe of the right lung, 80 cases (40.0%) in the lower lobe of the right lung, 60 cases (30.0%) in the lower lobe of the left lung, 30 cases (15.0%) in the upper lobe of the right lung, 20 cases (10.0%) in the upper lobe of the left lung, and 10 cases (5.0%) in the middle lobe of the right lung.

### 3.2. Diagnostic Results and Images of Chest CT

#### 3.2.1. Diagnostic Results of Chest CT

Among the 200 cases of preoperative CT, 196 cases (98.00%) showed the lesion and were clearly diagnosed, and 4 cases were missed.

#### 3.2.2. Chest CT Image

According to the main imaging findings of the lesions were as follows: (1) single large cyst (6.00%) showed single diameter >2 cm thin-walled cyst, with or without internal thin-walled separation. (2) The multiple large cysts (126 gamma 200∼63.00%) showed several regular or irregular large cysts (diameter > 2 cm) with multiple small cysts or microcysts of different sizes, which were arranged adjacent to each other. Thin line-like separation could be seen in the larger cyst lumen, and the largest cyst was about 13.7 cm in diameter. The intercystic lung tissue showed emphysema in 16 cases and localized emphysema in 6 cases. (3) Multiple cysts (21.00%) showed tight arrangement of thin-walled cysts with similar size of ≤2 cm, and honeycomb-like microcysts were shown in 6 cases. 4 patchy high-density shadows (16 gamma 200) 8.33%: on CT plain scan, the lesions showed smooth or nonsmooth patchy high-density shadow, with or without surrounding small gaseous cysts, and showed inhomogeneous enhancement, irregular cyst-like enhancement in 3 cases, and multiple round cyst-like enhancement in 6 cases. Refer to Figures 1–3.

### 3.3. Diagnostic Results and Images of LUS

#### 3.3.1. LUS Diagnosis Result

Of the 200 cases of preoperative LUS, 193 cases (96.50%) suggested the lesion and were clearly diagnosed, and 7 cases were missed.

#### 3.3.2. CPAM LUS Images of Children before Operation

The main LUS findings of children with CPAM were as follows: Figure 4: right congenital cystic adenoid malformation of the lung, CT revealed multilocular cystic lesions in the middle and lower lobe of the right lung, cystic adenomatoid malformation (type II), irregular hypoechoic consolidation area in the middle and lower lobe of the right lung, unsmooth and unclear pleural line, decrease or disappearance of A-line, dense B-line, or B-line fusion. Refer to Figures 4–9.

#### 3.3.3. CPAM LUS Images of Children after Operation

The boundary is not clear and the internal echo is uneven. No abnormal echo was found after operation. Refer to Figures 10 and 11.

### 3.4. CXR Diagnostic Results and Images

Among the 200 cases of preoperative chest X-ray, only 102 cases (51.00%) showed lesions, but all of them were not clearly diagnosed, 98 cases were misdiagnosed, of which 23 cases were diagnosed as normal chest film, 20 cases were diagnosed as increased texture of both lungs or inflammation of both lungs, retrospective analysis of 55 cases of missed chest X-ray was done, and lesions could be found in all cases, showing flaky increased brightness shadow in 25 cases and irregular blurred shadow in 20 cases. Refer to Figures 12–15.

### 3.5. LUS and CXR Check Results

Compared with postnatal chest CT, there was no significant difference in direct signs (including single or multiple cystic lesions) between LUS and CXR, but the indirect signs of LUS were significantly higher than those of CXR, and the difference between groups was statistically significant (*P* < 0.05). All the data results are shown in Tables 1 and 2.

### 3.6. LUS and CXR Check Results

The design route of this study was shown in Figure 16.

## 4. Discussion

CPAM belongs to a kind of congenital chest malformation in children, which is not uncommon in childhood malformations [8]. Due to the popularity of prenatal diagnosis, most CPAM can be found prenatal, and it is estimated that the actual incidence is much higher. In 2002, it was divided into 4 types according to tissue origin: type 0, large solid interstitial tissue of bronchial origin, also known as acinar dysplasia, most of the dead fetus could not survive; type 1, bronchial/bronchiolar source, diameter ≥ 2 cm large sac; type 2, bronchiolar source, a large number of vesicles; type 3, bronchiolar trachea/alveolar source, solid tissue; type 4, peripheral source, most large single cyst. In the new classification, types 0 and 3 were not cystic structure, and types 1, 2, and 4 had no adenoma. A retrospective study showed that the prenatal diagnosis rate of CPAM was 85.7%, and the average diagnosis time was 21–24 weeks of pregnancy [9]. Prenatal ultrasound needs to determine the size, location, and morphological characteristics of the mass, such as large, small, solid, or mixed, as well as changes in size and source of blood supply. The prenatal ultrasound of CPAM can be divided into three types: type I (about 25% of cases) is single or polycystic of different sizes, with a maximum diameter of 10 cm; type II (about 25% of cases) is mixed with cyst and surrounding tissue, and ultrasound echo is enhanced; type III (about 50% of cases) contains microcystic masses ≤5 mm [3]. The sensitivity and specificity of prenatal ultrasound are 90% and 77%, respectively. Most congenital malformations can be found by prenatal MRI [8]. The sensitivity and specificity of MRI diagnosis of pulmonary malformations are more than 95%. However, the advantage of MRI and ultrasound in diagnosis and prognosis is not obvious. MRI only has certain significance in complex or mixed cases [10, 11]. Once prenatal CPAM is found, it should be monitored regularly and attention should be paid to possible complications, such as mediastinal swing, fetal edema, and polyhydramnios. Daddi et al. [12] used ultrasonic measurement of CPAM volume ratio (CCVR) as an index to predict risk; if CVR > 1.6, there is an 80% risk of fetal edema [13]. If CVR > 0.84, the probability of severe respiratory distress caused by polyhydramnios and ascites will increase [14]. Other indicators include MRI lung volume, ultrasound ratio, and lung-to-head ratio, the main purpose of which is to monitor complications that may endanger fetal life [14].

Prenatal CPAM found that 70% of the children were found to be asymptomatic at birth, 30% of them had respiratory distress at birth, and 10% of them had severe respiratory distress requiring mechanical ventilation [15]. Fetal treatment includes glucocorticoid, minimally invasive, and fetal surgery [15]. For microencapsulated fetal edema, glucocorticoid therapy is more effective and less risky than open fetal surgery [15, 16]. The role of hormones is to reduce the production of fluid in the lungs and increase absorption, similar to the pathological changes in the later stage of the embryo. There were 3 cases of successful percutaneous sclerotherapy for type 2 and 3 CPAM. Catheterization in the thoracic cavity of the fetus with large sacs can be used for both diagnosis and treatment of fetal edema. Due to the reaccumulation of fluid after catheterization, a better method is to use pleural amniotic shunt. In cases where lung development is completed in the third trimester and giant cysts lead to mediastinal swing, termination of pregnancy can be considered for immediate postpartum treatment. Induced labor is considered only for fetuses with no hope of treatment. Most of the cases without prenatal diagnosis were found with CPAM after the occurrence of pneumonia, and 1 case with prenatal diagnosis of CPAM had respiratory symptoms at 1 month after birth [9]. The positive rates of CPAM diagnosed by X-ray and CT were 50% and 100%, respectively. Large cysts can lead to displacement of the trachea and mediastinum. Abnormal blood vessels should be observed for enhanced CT. Differential diagnosis should include pulmonary sequestration, congenital lobar emphysema, and bronchogenic cyst. It is difficult to distinguish PPB from type 4 CPAM imaging, and finally pathological diagnosis is needed. The timing of CT examination for prenatal diagnosis of CPAM and asymptomatic children after birth is still controversial. Some suggest that enhanced CT should be done before 6 months, and some should be completed before operation [17–20].

There is a consensus on surgical treatment for children with symptoms. There is no consensus on whether asymptomatic children need surgery. The reasons for supporting surgery are as follows: (1) infection during the observation period will increase the difficulty of operation and postoperative complications; (2) the nature of the tumor cannot be determined by imaging alone, especially the risk of pneumothorax, especially tension pneumothorax, between PPB and type 1 and 4 CPAM; (3) there is a risk of pneumothorax, especially tension pneumothorax; (4) some cases have the tendency of malignant transformation. It does not support the view of asymptomatic surgery: some cases have a tendency of degeneration, and surgery will increase the possible complications. It has been reported that 52 of the 90 cases received conservative treatment without obvious symptoms [21]. In detail, 20% of asymptomatic children develop symptoms, and a retrospective survey found that 45 infants underwent surgery after symptoms, with an increase in intraoperative and postoperative complications compared with asymptomatic surgery [22]. The earlier the operation, the more beneficial to the development of the residual lung, which is also one of the reasons to support the early operation. At present, it is generally accepted whether to choose the operation and the best time should consider the following factors: (1) the space-occupying effect and symptoms of the cyst; (2) the requirements of the parents; (3) the evaluation of the anesthesiologist; (4) the experience of the surgeon. At present, the age of asymptomatic children undergoing surgery in China is from 6 months to 1 year. In the past, the standard operation was thoracotomy, but video-assisted thoracoscopy has become a widely accepted operation in recent years. In the United States, the proportion of video-assisted thoracoscopy is gradually increasing, and compared with thoracotomy, postoperative complications and hospital stay are similar [23]. Meta-analysis unveiled that the complications after thoracoscopic surgery were reduced, and the hospitalization time was shortened, but the operation time was relatively prolonged [24]. Video-assisted thoracoscopic surgery requires one-lung ventilation to provide sufficient surgical space for the collapse of the lung on the affected side and low CO2 pressure if necessary, with the cooperation of an experienced anesthesiologist. If thoracotomy is performed, it is best to use the muscle pull approach to avoid damage to the anterior patellar muscle, latissimus dorsi, and its nerves and to reduce postoperative pain and muscle atrophy. In the neonatal period, video-assisted thoracoscopic surgery is more difficult because of the small surgical space. But for newborns under 3 months old, video-assisted thoracoscopic surgery in experienced medical centers is also safe and effective, with a thoracotomy rate of between 3% and 12.2% [25]. The choice of lobectomy or partial lobectomy depends on whether to remove the lesion completely or to preserve healthy lung tissue as much as possible. Lobectomy is a standard operation, and partial lobectomy has been increasing in recent years because some lesions do not involve the whole lobe of the lung. Partial resection includes anatomical segmental resection, wedge resection, and nonanatomical segmental resection [25]. The benefit of lobectomy lies in the complete removal of the focus, no residue, avoiding the deterioration of the residual focus, and reducing postoperative air leakage. The operation space in the chest of children is small, and the more complex the local resection is, the more difficult it is. The recovery time after partial lobectomy is longer than that after lobectomy [26]. Video-assisted thoracoscopy cannot touch the boundary of the mass by hand, and it is difficult to determine with the naked eye, and it is difficult to avoid residual lesions after partial resection. Unless multiple lesions involve several lobes, there is no definite basis for recommending partial resection, and local resection is only suitable for very limited lesions [25, 26]. CPAM is associated with two kinds of malignant tumors, one is PPB in infants or young children, and the other is bronchoalveolar carcinoma in adolescence or adults. Bronchoalveolar carcinoma and the characteristics of premolecular malignancy in type I CPAM mucin cells occurred in many cases without complete resection of CPAM, which confirmed the relationship between bronchoalveolar carcinoma and type I CPAM. Pleuropneumoblastoma is a rare chest tumor, which is mostly diagnosed before 6 years of age. It can be divided into three types: type I, cystic type, type II, mixed type, and type III, solid. The clinical manifestations are lack of specificity, only repeated pulmonary infection, unexplained pneumothorax, and nonspecific X-ray findings. Neither imaging nor biological markers can clearly distinguish type 1 PPB from type 4 CPAM [27]. Some patients were even diagnosed as CPAM before delivery and confirmed as PPB after operation. PPB should be highly suspected in patients with family history, infantile spontaneous pneumothorax, renal cyst, intestinal polyp, thyroid hyperplasia, and gonadal tumor. 40% of PPB can find relevant clues, and the prognosis of patients with early diagnosis of cystic PPB is significantly better than that of patients with solid tumors. The incidences of CPAM and PPB are 120000 and 1250000, respectively; that is, 4% of CPAM may be pleural PPB.

Chest X-ray is an important imaging examination of pulmonary diseases in children, but for rare diseases such as CPAM, chest X-ray has low specificity and low sensitivity, which may lead to missed diagnosis and misdiagnosis [28]. It is reported that the sensitivity of chest X-ray in the diagnosis of CPAM is only 61% [28]. In the current study, only 51.67% of the lesions are indicated, and there is no clear diagnosis. However, no definite diagnosis was made in 29 cases, of which 8 cases were diagnosed as normal chest X-ray, 10 cases were diagnosed as increased texture of both lungs or inflammation of both lungs, retrospective analysis of 14 cases of missed chest X-ray was done, the lesions were found in 6 cases, and irregular blurred shadow was found in 6 cases. In this group of cases, CPAM chest film showed localized transmittance increased shadow, flaky blurred shadow, or focal multiple small gas and fluid shadow, which was easily confused with pneumonia, diaphragmatic hernia, pneumothorax, and other congenital pulmonary cystic lesions. In contrast, CT is the best method for the diagnosis of CPAM, and its sensitivity and specificity are much higher than those of ultrasound, chest X-ray, and other examination methods. In the study of Jeong et al. [29], the sensitivity and specificity for CT diagnosis of CPAM were 93.3% and 93.7%, respectively. In this study, the detection rate of CPAM lesions was 98.33%, which was much higher than that of chest X-ray (51.67%). However, the diagnosis rate of the first diagnosis is only 70.6%. The retrospective diagnosis test reflects that there is a certain correlation between the understanding of the disease and the diagnostic efficiency. It can be inferred that the low diagnosis rate of this group of cases is mainly related to the lack of understanding of the disease in the past. By strengthening the understanding of CPAM, the diagnostic accuracy of CPAM can be improved. In the diagnosis and treatment of CPAM, for children with high risk, asymptomatic after birth, disappearance of thoracic mass in the third trimester of pregnancy, and children with CPAM in twins or multiple births, the postnatal differential diagnosis of CPAM mainly relies on traditional CXR and CT. CXR is the first choice for the diagnosis of CPAM after birth. Its manifestations include multiple focal low-density shadow, focal vesicular transparent shadow, focal hyperinflated or clouded mass in the lung, hyperventilation, mediastinal displacement, pneumothorax, and so on when the lesion is huge. However, postnatal examination based solely on CXR has great limitations, and the misdiagnosis rate is high. CT is the imaging standard for preoperative diagnosis of CPAM, but CT is radioactive and expensive, so it needs to be cooperated with children after the use of sedatives and often needs to be evaluated by chest CT. LUS has the advantages of simplicity, easy operation, strong repeatability, low cost, and less radiation. It is considered that LUS can accurately diagnose various lung diseases, and LUS is considered to be more accurate and sensitive than traditional CXR in the diagnosis of pneumothorax, pulmonary edema, pulmonary consolidation, and pleural effusion, avoiding repeated CT examination. Our study still has some shortcomings. Firstly, the quality of this study is limited due to the small sample size we included in the study. Secondly, this research is a single center study and our findings are subject to some degree of bias. Therefore, our results may differ from those of large-scale multicenter studies from other academic institutes. Our research is still clinically significant and further in-depth investigations will be carried out in the future.

In conclusion, the most common CT findings of CPAM in children are cystic lesions, especially polycystic lesions, while LUS images of CPAM in children are various. LUS is a noninvasive and nonradiological examination method, which is easy to operate and repeat. LUS can be used for preliminary qualitative screening of CPAM in children, and the diagnostic value of indirect signs of LUS is better than that of CXR (Figure 16).

## Figures and Tables

**Figure 1:** The brightness of the left lower lobe increased with a range of about 32.3 mm × 45.6 mm × 62.8 mm. The inner lung texture was sparse, with bronchovascular bundle running, no clear envelope at the edge, and no clear abnormal aortic blood supply. The remaining two lung fields were clear, lung texture was regular, and no abnormal tissue density shadow or space-occupying lesions were observed. Trachea and bronchus were unobstructed without stenosis or obstruction, and hilar shadow was not significant. No abnormal enhancement was found in both lungs on enhanced scan. The mediastinal structure was clear, no lesions were observed, and no enlarged lymph nodes were observed beside the trachea, under the carina, in front of the vessels, and behind the vena cava. There was no bilateral pleura thickening and no pleural effusion. Left lower lobe changes, considered congenital pulmonary airway malformation, cystadenoma malformation (type II).

**Figure 2:** Multiple cystic transparent shadows can be seen in the right lung field with a range of 57 × 68 × 68 mm and a clear boundary. The size of the inner capsule is different; the largest one is about 53 × 48 × 26 mm. A large amount of liquid density shadows can be seen in the lung, and the liquid-gas plane can be seen. The mediastinum pushes to the left, pressing the left lung. Patchy and slightly high-density shadows were seen in the lower lobe of the left lung, with less clear boundaries. No thickening of the left pleura, no effusion of the left pleura. 1. Abnormal changes in the right lung, considered congenital cystadenoma malformation of lung (type I). Mediastinal displacement was obvious and left lung was compressed. Left lower lobe consolidation with a few exudative lesions.

**Figure 3:** Multiple cystic lucid areas in the posterior segment of the upper lobe and lower lobe of the right lung, with a range of about 6.2 cm × 6.8 cm × 7.9 cm, were displaced to the left by mediastinal compression. Multiple patchy and cordlike fuzzy shadows were seen in both lungs, partial consolidation was seen in the right lung, and air bronchial shadows were seen inside. Trachea and bronchus were unobstructed without stenosis or obstruction, and hilar shadow was not significant. The mediastinal structure was clear, no lesions were observed, and no enlarged lymph nodes were observed beside the trachea, under the carina, in front of the vessels, and behind the vena cava. There was no bilateral pleura thickening and no pleural effusion. Cystadenoma malformation (type I) was considered.

**Figure 4:** Left congenital cystadenoma. CT showed increased transmittance of the posterior segment of the upper lobe and the dorsal segment of the lower lobe of the left lung, with a range of about 38.5 *∗* 26.6 *∗* 42.9 mm, with multiple round areas of different sizes, with a maximum diameter of about 7.7 mm, some of the walls slightly thicker, enhancement of the cyst wall, thickened pulmonary artery blood supply, and cystic adenomatoid malformation of the lung (type II). Ultrasound revealed irregular hypoechoic pulmonary consolidation areas, pleural lines were not smooth and unclear, A-lines decreased or disappeared, and dense B-lines or B-lines fused.

**Figure 5:** Right congenital cystic adenoid malformation of the lung, CT indicates abnormal changes of the right lung, considering congenital cystic adenomatoid malformation (type I); multiple cystic transparent shadow can be seen in the right lung field, the range is about 57 × 68 × 68 mm, the boundary is clear, the size of the internal capsule is different, the largest is about 53 × 48 × 26 mm, a large amount of fluid density shadow can be seen in it, the liquid-gas plane can be seen, and a little normal lung tissue can be seen near the middle lobe of the right lung. Ultrasound revealed a huge cystic echo in the right lung.

**Figure 6:** Ultrasound indicates irregular hyperechoic or mixed echo areas.

**Figure 7:** Ultrasound indicates irregular hyperechoic or mixed echo areas.

**Figure 8:** Ultrasound indicates irregular hyperechoic or mixed echo areas.

**Figure 9:** An irregular mixed echo mass can be seen in the right lung field, mainly solid, the size is about 71 *∗* 51 *∗* 47 mm, the boundary is not clear, the irregular anechoic area can be seen inside, and the largest is about 20.9 *∗* 10.4 mm. The left lung field was obviously squeezed and shifted to the left.

**Figure 10:** An irregular hyperechoic area can be seen in the upper part of the left lung field.

**Figure 11:** The pleural line of the bilateral lung field was smooth, the lung was slippery, the echo distribution of the lung field was uneven, part of the A-line disappeared, and there was no obvious abnormal mass echo and pleural effusion.

**Figure 12:** Both sides of the thorax are symmetrical, and the bones of the thorax are complete. The distribution of lung markings in both lungs is regular, with clear borders, and no signs of pulmonary congestion or congestion; both lung fields are clear, with no lung parenchyma or interstitial lesions; bilateral hilar size, shape, and location are not abnormal; no mediastinal widened.

**Figure 13:** Both sides of the thorax are symmetrical, and the bones of the thorax are complete. The distribution of lung markings in both lungs is regular, with clear borders, and no signs of pulmonary congestion or congestion; both lung fields are clear, with no lung parenchyma or interstitial lesions; bilateral hilar size, shape, and location are not abnormal; no mediastinal widened.

**Figure 14:** The right thorax was slightly full, and the right lung transparency was increased. Multiple cystic translucent areas were seen in the right middle and lower lung fields, with an area of about 46 × 67 mm, and the boundary was not clear. The lung markings of the left lung increased and thickened, and a few patchy blurred shadows were seen in both lungs, especially in the lower left lung, and the size, shape, and position of the left hilum were not abnormal; the trachea, mediastinum, and heart shadows shifted slightly to the left. The mediastinum was not widened. Consider cystadenoma malformation (type I).

**Figure 15:** Both sides of the thorax are symmetrical, and the bones of the thorax are complete. In the right lower lung field, there was a local increase in transparency, and the lung texture was disordered, with a range of about 24 × 25 mm; the distribution of the lung texture in the other two lungs was regular, the edge was clear, and no signs of pulmonary congestion or congestion were found; the size, shape, and location of the bilateral hilum were unknown. See abnormal; no mediastinal enlargement.

**Figure 16:** Research route.

**Table 1:** Comparison of direct and indirect signs between 1LUS and CXR [*n*/%].

Grouping	*N*	Direct sign	Indirect sign
LUS group	200	82 (41.00)	200 (100.00)
CXR group	200	80 (40.00)	86 (43.00)
*χ* ^*2*^		0.041	**159.440**
*P*		0.838	**0.000**

It is statistically significant that bold values are used to highlight differences.

**Table 2:** Comparison of indirect signs between pulmonary X-ray and pulmonary ultrasound [*n*/%].

Grouping	*N*	Pulmonary consolidation	Mediastinal displacement	Pleural effusion	Bronchial aeration	*A*-line	*B*-line	Pleural line	Exudative lesion
LUS group	200	132 (66.00)	120 (60.00)	6 (3.00)	80 (40.00)	186 (93.00)	200 (100.00)	182 (91.00)	—
CXR group	200	90 (45.00)	120 (60.00)	0 (0.00)	—	—	—	—	86 (43.00)
*χ* ^*2*^		17.856	0.000	0.616	—	—	—	—	—
*P*		**0.000**	1.000	0.947	—	—	—	—	—

It is statistically significant that bold values are used to highlight differences.

## Data Availability

The datasets used and analyzed during the current study are available from the corresponding author upon reasonable request.
